# Study on the Impact of Online Courses for Pregnant and Lying-In Women on Maternal and Infant Health during the Epidemic

**DOI:** 10.1155/2021/4019210

**Published:** 2021-12-20

**Authors:** Liangfang Shi, Ling Yuan, Lin Zhou, Shuixian Zhang, Xia Lei

**Affiliations:** Department of Obstetrics, Affiliated Hangzhou First People's Hospital, Zhejiang University School of Medicine, Zhejiang, Hangzhou 310006, China

## Abstract

The sudden outbreak of the new crown pneumonia has brought online learning from a supporting role to the center of the teaching stage in an instant. On the basis of the feasibility analysis and demand analysis of the microcourse learning system, this paper uses Sina cloud server to build the WeChat public platform learning online course and designs and implements the microcourse learning system function based on the microcourse public platform. We completed the recording, editing, publishing, and testing of microclass courses and provided services for teachers and pregnant women's microclass learning in order to achieve better learning results. A total of 151 people regularly participate in maternity school courses, accounting for 30.4%. There are 190 people who have never attended the maternity school course, accounting for 38.2%. There are 156 people who occasionally participate in maternity school courses, accounting for 31.4%. The top five sources of health information during pregnancy are books, maternity schools, experience of elders, the Internet, and television. The results of one-way analysis of variance showed that pregnant women of different ages had statistically different scores in the dimensions of knowledge and ideas (*P* < 0.05). There are statistical differences in the scores of pregnant women with different economic incomes in this dimension (*P* < 0.05). The women with economic income ≥5000 yuan/month have the highest scores, and those with economic income ≥5000 yuan/month have the lowest scores. The scores of pregnant women who participated in the maternity school were significantly higher than those who did not participate in the maternity school (*P* < 0.05). There are statistical differences in the scores of maternal and child health basic skills among pregnant women of different age groups (*P* < 0.05). The women aged ≥35 years old have the highest scores, and those aged 20–24 years old have the lowest scores. The differences in the scores of pregnant women with different economic incomes in this dimension are statistically significant (*P*＜0.05). The women with economic income ≥5000 yuan/month have the highest score, and those with economic income<2000 yuan/month have the lowest score. Participation in maternity schools has an impact on the scores of this dimension. Pregnant women who regularly participate in maternity schools have the highest average scores, and those who do not participate in maternity schools have the lowest average scores.

## 1. Introduction

Since December, 2019, a new type of coronavirus infection pneumonia has broken out in our country [1]. The online teaching setoff under the background of “stopping classes and not stopping school” has brought “rare” development opportunities for the promotion of teaching reform in the era of “Internet + education”, renewing teaching concepts and innovative teaching methods, as well as many severe challenges [2]. In order to ensure that pregnant women can carry out online learning at home, some teachers use online course platforms for asynchronous course teaching, some teachers use live broadcast tools or video conference tools for live synchronous teaching, and some teachers use WeChat groups for instant interactive teaching. It is undeniable that diversified media tools provide many feasible solutions to the problem of time-space separation between teachers and students in online teaching. However, on the one hand, because the online teaching programs formulated by some local education administrative departments have not been widely used, many teachers mistakenly believe that online teaching is “traditional classroom online moving”, resulting in a simplification of online teaching methods. Fully online teaching is prone to low learning input and low satisfaction among pregnant women, which arouses reflections from managers and teachers. How to help teachers recognize and understand online teaching and how to organize and carry out online teaching efficiently has become a problem we must face [3].

Due to the continuous updating of the concept of childbirth and the lack of childbirth experience of primiparas, primiparas have an urgent need for health education knowledge before, during, and after delivery [4]. Pregnant women's school is a fixed place for prenatal health education. Routine prenatal health education is conducted in groups of pregnant women's schools, issuing health education manuals, taught by full-time teachers, and recorded by the mothers, and the teaching time is mostly carried out on working days. Because each primipara has a different understanding of perinatal knowledge, in the traditional health education model of maternity school group teaching, there is a real problem that full-time teachers give lectures in class, and primiparas cannot keep up with the rhythm [5]. As time goes by, primiparas will have more and more doubts about prenatal health education knowledge. The traditional mode of teaching in groups for pregnant women is at a fixed time, and most of them are taught on weekdays. Primiparous women cannot attend classes in time due to work and other reasons, which will affect the learning effect, fail to achieve the expected goal of prenatal health education, and affect the treatment effect and patient satisfaction. The traditional prenatal health education model can no longer fully meet the needs of primiparous women for prenatal health education knowledge [6, 7]. Therefore, it is particularly important to explore the prenatal health education model combined with Internet technology.

This article has completed the feasibility analysis and demand analysis of the microcourse learning system and analyzed and designed the microcourse curriculum. The main content of this article is the design and implementation of a microcourse learning system based on the WeChat official account, which mainly includes the design and implementation of the WeChat terminal and background management system. We record and edit the microclass curriculum and publish the microclass curriculum to the microclass learning system after the microclass production is completed. Combining the relevant functions and modules of the WeChat official account design, it is convenient for teachers and pregnant women to better use the microclass courses for learning. The results of multivariate analysis showed that age and attendance of pregnant women's school were the influencing factors of maternal and child health literacy qualifications of pregnant and lying-in women. Pregnant and lying-in women have a better grasp of basic skills and have a poorer understanding of lifestyle and behavior. Age, economic income, and attendance of maternal school may be the influencing factors of the scores of maternal knowledge and ideas.

## 2. Related Work

In recent years, with the vigorous development of microvideo, research on the background, development and prospects, current situation and problems, design and application of microvideo has become a hot spot for domestic scholars [8]. Specifically, microvideos are used for network communication. Scholars believe that microvideo can be used as a way of spreading news and events on the Internet and has an important position in the era of mobile Internet [9]. The advantages of video resources can satisfy users who are not limited by time and space and can watch the resources they need. Through the research and analysis of the current situation, problems and solutions of the microvideo development, the content construction, operation mode, resource integration, and other aspects of the microvideo website are discussed.

Regarding the application of microvideo to education and teaching, most scholars study the application of microvideo in specific disciplines, as well as the application in distance education and training. In addition, the application research of microvideo in informal learning is also a hot issue. With the theoretical support of mobile learning, microlearning, ubiquitous learning, fragmented learning, informal learning, etc. and the background of the times, microvideo has been widely used in many fields due to its short, precise, and fast characteristics. Research on the application of microvideos in different fields has also been showing an upward trend. The fields and research related to this research include microvideo design research in family counseling for children, research on the production and application of nursing videos for pregnant women and newborn babies, and research on pediatric nursing training and teaching based on microvideo technology. However, there are relatively few researches on the design and development of mobile learning resources for microvideos for mothers and babies.

In terms of education and teaching, Youku has a very close cooperation with the Massachusetts Institute of Technology in the United States. The school unconditionally uploads excellent teaching courses and resources to the Youku network to facilitate independent learning by pregnant women. The foreign education field has brought a huge impact and has brought a good start to the equalization of educational resources relying on the Internet [10]. With the open sharing of Internet resources, microvideo learning resources have been used by more and more people from all walks of life, so that learners can enjoy without the restrictions of the network, education level, regional differences, time, space, etc. These excellent microvideo course resources promote the change and development of people's learning and life and play an important role in education fairness, social harmony, and improving people's happiness [11].

The study found that the proportion of pregnant women with various health literacy is less than 50%, but the correct answer rate for some common infectious diseases to be checked and prevented for the first prenatal check-up is higher, which is more in line with the promotion of the prevention and control of infectious diseases [12]. However, other maternal and child health care knowledge is not relevant enough. Related scholars' research on the current status of maternal health in Wuhan found that the cesarean section rate in Wuhan rose from 46.26% in 2003 to 65.28% in 2008, and it has shown an upward trend in recent years [13]. There are many reasons for the increase in the cesarean section rate, and the subjective wishes of pregnant women play a big role, which may be related to their level of health literacy. Relevant scholars conducted a survey on the health literacy status of mothers and infants among 1,800 participants who participated in health education activities in Haidian District, Beijing [14]. The results found that the survey participants had the highest awareness of mothers' basic knowledge, which shows that pregnant women pay more attention to their own health care. Research shows that prenatal health education for primiparas based on flipped classrooms can improve the self-efficacy of childbirth, breastfeeding self-efficacy, and maternal and infant health literacy of primiparas and is an effective way to carry out prenatal health education for pregnant women [15]. However, its research only implemented prenatal health education in the flipped classroom model at 36 to 39 weeks of gestation and did not systematically design the prenatal health education program, so its results cannot fully reflect the effect of the implementation of prenatal health education for primiparas.

Studies have found that the level of health literacy of women in New York is related to whether they can correctly understand prescriptions and drug instructions and use them correctly [16]. Studies have shown that pregnant women of different races have different levels of knowledge about health literacy [17]. 8% of black women still smoke during pregnancy, while the proportion of whites is as high as 34%. Many people do not know enough about the extent to which smoking harms the fetus. Relevant scholars found in a study that 16% of women have a low level of education, 61% of women start antenatal care three months after pregnancy, and 50% of the survey subjects underutilize antenatal care [18]. Researchers' cross-sectional study of pregnant women in rural India showed that the utilization rate of health care services among survey respondents was low, and there was no difference in utilization rates among survey respondents of different social status [19]. A current status study conducted by related scholars on pregnant women found that more than 40% of the 2257 study subjects did not supplement iron intake as required. The study showed that there is a need to increase iron supplement coverage for pregnant women, especially those who are considered high-risk pregnancy [20]. The longevity of Japanese people is supported by data, which has a nonnegligible relationship with their good health status. In the field of maternal and child public health, Japan has implemented a folic acid supplement program to reduce neural tube defects in newborns.

## 3. Social Support Analysis of WeChat Parenting Group Users

### 3.1. Obtain Information to Support Self-Empowerment

Information support refers to providing suggestions and guidance to the other party that help solve problems. The traditional offline social support system can provide pregnant women with sufficient emotional support and substantial support, but they cannot provide them with sufficient parenting information support.

Due to advances in technology, the information obtained from the online parenting community is often updated faster than the information provided by offline professional health care workers and relatives of pregnant women. Compared with family members, there is a weak relationship between pregnant women and members of the online parenting community. As the main offline information support source, the female relatives of pregnant women have many similarities with their own backgrounds and experiences. They can provide parenting support, but they tend to be homogeneous, and the amount of useful information is not large. However, due to the greater differences in knowledge structure, experience, background, etc. among members in the online parenting community, the information exchange between each other is more diversified.  Figure 1 shows the changes in social support received by WeChat parenting group users.

In the new era, young women use the Internet to obtain information support in various ways. They can obtain existing information from traditional Internet search engines to forums, and they can also obtain online information support through social network media. The role of social networks in supporting information after women give birth is particularly important. It is worth noting that these pregnant and lying-in women are wary of the fact that the unevenness of parenting information on the Internet will also confuse searchers. At the same time, there are differences in the level of Internet use by users. Therefore, there are individual differences in the level of cognition and discrimination of information on the Internet, and users need to improve their own efficiency to distinguish, learn, and respond to this information.

In the process of pregnant women using WeChat groups to improve self-empowerment, practical information is often the fastest and most effective. In online parenting groups, what is most needed every day is often this kind of information. Even some group members will provide a lot of parenting knowledge without anyone asking. During the outbreak of vaccine issues, members of the group will share new developments in vaccine reports every day. In addition, information on discounts at major online and offline shopping malls is also useful and frequently discussed information regarding future employment.

The strong interactivity in the WeChat group is also a necessary reason for pregnant women to complete their self-empowerment. The online parenting group observed this time has more than 100 members, who speak a lot every day, and often chat messages in one day reach 999+. Whether it is consultation or answer, the speech of group members will drive the next wave of interaction within the group. For example, when a group member indicated that they wanted to go to a newly opened mall, several group members immediately asked them to share the new store and new discount information of the mall. The members of the group also used multimedia to give detailed explanations of the mall from pictures to videos, to voices, to texts, and even attached specific locations and transportation methods. Then the group members continued to ask questions, and the group members continued to answer.

### 3.2. Obtaining Companion Support and Conversion of Online and Offline Relationships

Companionship support refers to the support when an individual spends time with others to provide personal relaxation or entertainment and help others reduce stress. Although the WeChat parenting group is a weakly connected group, group members often accompany each other during pregnancy. Many mothers will tell everyone in this group before giving birth, and people in the group will also accompany them online. Although they cannot accompany them like offline relationships, they can accompany them regardless of time and place online, and they will not be unable to accompany them because of geographic distance.

Although this group does not discuss much about the content of work at work, and a certain percentage of mothers are recuperating at this time, there are still enthusiastic group members who make suggestions. When group members encounter the embarrassing situation of breastfeeding and cannot communicate with colleagues, group members can also achieve online “cloud accompany” to comfort and provide support to the parties in time and sometimes even enlighten the parties with their previous experiences and ease them.

In addition, there are not a few people who transform online relationships into offline relationships. Sometimes it was for the purpose of trading second-hand items and sometimes because the place of residence was close, and online group members met offline. After getting acquainted with each other, the members of the group will also meet to go shopping together, gather together, play mahjong together, and go to beautify together. Group members who are acquainted with each other even talk about baby kisses with a smile after seeing each other's babies.

## 4. Design of the Online Microcourse Learning System for Pregnant and Lying-In Women

### 4.1. WeChat Official Account Learning Network Online Course Development Model

Considering the needs of microcourse courses, this study uses the subscription number in the WeChat official account. In terms of microcourse teaching, the subscription number has some advantages compared with the service account and the enterprise account. To meet the needs of microcourse courses, it is convenient for teachers to share teaching resources with learners through WeChat public accounts.

The WeChat official platform provides an editing mode and a development mode. The two modes are mutually exclusive and cannot be opened at the same time, but they can be switched at any time. The development mode of the micro official account is not open to all users. The official account cannot be used for the development of high-end interfaces. The development of high-end interfaces can only be carried out after passing WeChat authentication. There are three authentication methods: legal representative authentication, payment authentication, and WeChat authentication. After the WeChat subscription account authentication is completed, we can enter the development mode of WeChat. The developer mode of WeChat includes four modules, namely basic configuration, developer tools, operation and maintenance center, and interface permissions. After entering the development mode, open the developer password and fill in the server configuration information.

#### 4.1.1. Server URL Access

WeChat public platform needs to do some preparatory work between development, mainly about the configuration of the server address (URL) and the verification of the token because we must first ensure that the server is in the public network environment to ensure that the WeChat server can be accessed. Common public network servers include Sina Cloud and Baidu Cloud. The public network server selected in this study is Sina Cloud Server.

#### 4.1.2. Data Exchange Method

After the WeChat public platform successfully connects to the website, the developer can obtain the authority of the message interface, and the message interface provides developers with the function of communicating with users. When a WeChat user sends a message to the WeChat official account via WeChat, the WeChat server will send the message to the developer's URL. When the URL receives the message, after parsing and classifying the message, the content that needs to be replied is returned to the WeChat server, and the WeChat server replies the returned message to the WeChat user.

### 4.2. The Overall Architecture Design of the System

Figure 2 shows the overall architecture diagram and specific system functions and characteristics of the microcourse learning system based on WeChat public.

#### 4.2.1. Basic Layer

The construction of the basic layer of the system is the basis for the construction of the system. The basic layer of this research includes two parts: physical facilities and IaaS. The physical facility layer includes servers, storage, and network parts. IaaS mainly refers to virtual servers. The server mainly relies on Sina Cloud to support the application requirements of the learning system to meet the needs of WeChat users.

#### 4.2.2. Data Layer

The data layer of the microcourse learning system mainly manages the information of WeChat users, including the storage, processing, and exchange of user information in order to better manage user information.

#### 4.2.3. Service Layer

It mainly includes system management services, data analysis services, and task handling services. This article mainly connects the WeChat official platform through the WeChat platform server to provide services for learners who are concerned about the WeChat official account.

#### 4.2.4. Exchange Layer

The exchange layer of the microcourse learning system mainly connects the service layer and the application layer. It mainly includes two parts: a message bus and an interface service. The message bus transmits asynchronous messages to the application layer.

#### 4.2.5. Application Layer

The system application layer is the presentation layer of the system construction. The microcourse learning system mainly provides various application modules provided by the system to teachers and learners. These modules provide course information and related services to learners and teachers.

#### 4.2.6. User Layer

The user layer of the system is the experience layer constructed by the system. The user layer of the microcourse learning system mainly provides services for the users of the WeChat official account.

### 4.3. System Function Module Design

The front-end WeChat front-end is convenient for managers of WeChat official accounts to manage teaching resources and users' personal information.

#### 4.3.1. Front-End Module Design

Figure 3 shows the functional schematic diagram of the microcourse learning system based on the WeChat official account. The three modules of the microcourse learning system can basically meet the curriculum needs of learners and teachers. In addition, the microcourse learning system has designed relevant submodules according to the needs of users to enable learners to achieve better learning results.

#### 4.3.2. Back-End Module Design

With the help of the WeChat public platform, teachers can easily complete the management operations of the microcourse learning content without the help of administrators and send relevant information and course content by themselves. The back-end management based on the microcourse learning system is the guarantee for the front-end operation of WeChat, which mainly includes two parts: user management and resource management.

The user management module mainly includes two submodules, user information and user authority. User information includes teachers and maternal users. Users who follow the WeChat official account can use this module to improve and modify their information. The user authority module mainly sets different authority for teachers and learners through the WeChat public platform. The authority of the teacher user is higher than that of the learner user, which is convenient for better management of microcourse teaching to achieve better teaching effect.

The resource management module mainly includes two submodules: message management and course management. Message management means that teachers use the WeChat public platform to group and send messages to users who follow the WeChat official account according to the learner's different learning conditions, and learners use this module to feed back the problems encountered in learning to teachers in a timely manner. The course management module is for teachers to manage course information through the WeChat public platform, which mainly includes the classification, uploading, and replacement of course resources, so as to better serve the microcourse learning system.

### 4.4. Evaluation of the Impact of Online Courses on Maternal and Infant Health

It is generally measured from three aspects: consistency, monotonicity, and accuracy. Among them, consistency means that the error of the designed evaluation algorithm under different test samples is as small as possible, that is to say, the evaluation algorithm should be widely used; monotonicity refers to the change rule of the evaluation value of the designed evaluation algorithm and the subjective evaluation value. Accuracy means that the error between the evaluation value of the designed evaluation algorithm and the subjective evaluation value should be as small as possible. Here are a few more commonly used mathematical evaluation indicators:

(1) The formula of Spearman rank ordered correlation Coefficient (SROCC) is as follows:
  (1) $$\begin{array}{c} \text{SROOC}=1-\frac{\prod_{i=0}^{n-1}{\left(r_{xi}-r_{yi}\right)}^{2}}{\left(n-1\right)\left(n-2\right)}. \end{array}$$
Among them, *r*_*xi*_ and *r*_*yi*_ are the sorting positions of the corresponding sequence of *x* and *y*, respectively, and *n* is the number of samples tested.
(2) Linear Pearson Correlation Coefficient (LPCC) formula is as follows:
  (2) $$\begin{array}{c} \text{LPCC}=\frac{\prod_{i}\left(s_{i}-\overset{⌢}{s}\right)•\left(s_{pi}-{\overset{⌢}{s}}_{p}\right)}{\sqrt{\prod_{i}{\left(s_{i}-\overset{⌢}{s}\right)}^{2}}•\sqrt{\prod_{i}{\left(s_{pi}-{\overset{⌢}{s}}_{p}\right)}^{2}}}. \end{array}$$
Among them, *s_i_* represents the subjective score, and *s_p_* represents the image quality prediction score based on the regression function.
(3) Kullback-Leibler divergence (KLD), also known as KL distance and relative entropy, is used to measure the difference in the distribution of two probability density functions. The algorithm formula is as follows:
  (3) $$\begin{array}{c} \text{KLD}\left(\frac{p}{q}\right)=\prod_{i}p\left(i\right)\log\left[\frac{q\left(i\right)}{p\left(i+1\right)}\right]. \end{array}$$
Among them, *p* represents the true histogram mapping generated by the probability density function, and *q* represents the predicted histogram mapping generated by the probability density function.
(4) The formula of Outlier Ratio (OR) is as follows:
  (4) $$\begin{array}{c} \text{OR}=\frac{\gamma }{\Gamma }. \end{array}$$
Among them, *γ* represents the number that exceeds the subjective score by 2 standard deviations, and Г represents the total number of participants in the predictive evaluation.
(5) The formula of Outlier Distance (OD) is as follows:
  (5) $$\begin{array}{c} \text{OD}=\underset{i⟶I_{f}}{\prod }\min\left[s\left(i\right)-f\left(i\right)-2\delta_{s}s\left(i\right)+2f\left(i\right)-2\delta_{s}\right]. \end{array}$$

Among them, *I_f_* represents the set of outliers, *s*(*i*) represents the DMOS or MOS value of image *i*, and *f*(*i*) is the predicted value after logical transformation. The logical transformation formula is as follows:

(6) $$\begin{array}{c} f\left(x\right)=\frac{\theta_{1}-\theta_{2}}{1-\exp\left(x-\theta_{3}/\theta_{4}\right)}-\theta_{2}. \end{array}$$

Among them, *θ*_1_, *θ*_2_, *θ*_3,_ and *θ*_4_ are model parameters selected from the minimum mean square error between the predicted value and the subjective value.

## 5. Results and Analysis

### 5.1. Prenatal Education Received by Pregnant Women

Pregnant women who have participated in all courses of the maternity school are defined as regular attendance, and women who have participated but have not participated in all courses are defined as occasional attendance. Among the 800 pregnant women surveyed, the number of women who were able to regularly participate in maternity school courses was the least, with a total of 100 women, accounting for 12.5%. The number of people who have never participated in maternity school courses is the largest, with a total of 500 people, accounting for 62.5%. There are 200 people who occasionally attend the maternity school courses, accounting for 25%. This shows that the proportion of pregnant women receiving formal prenatal education is relatively low, and the penetration rate of pregnant women's schools needs to be increased. See Table 1 for the participation of pregnant women in school education for pregnant women.

A survey of the sources of health information received by pregnant women during pregnancy found that, in descending order of the number of people, they were online courses, books, pregnant women's schools, elders' experience, Internet, television, and medical staff.  Figure 4 shows the sources of health information for pregnant women during pregnancy.

### 5.2. Awareness of Maternal Knowledge and Concepts and Analysis of Influencing Factors

A survey on the awareness of pregnant women's knowledge and concept dimensions found that the highest awareness rate is “understanding the dangers of diet, nutritional requirements and smoking, drug abuse and alcohol abuse in the third trimester of pregnancy” to the fetus. 474 of the 497 pregnant women said they were aware of it. The awareness rate was 95.37%. Followed by “knowing the benefits of breastfeeding”, 466 pregnant women said they were aware; the awareness rate was 93.76%. The item with the third awareness rate is “normal fetal heart sounds are 110–160 beats/min.” There are 434 pregnant and lying-in women expressing awareness, and the awareness rate is 87.32%. The item with the lowest awareness rate is “knowing the time of the first antenatal check-up”. Only 241 pregnant women said they knew it, and the awareness rate was 48.49%. The knowledge and concept awareness of 800 pregnant women are shown in Figure 5.

A one-way analysis of variance was performed on the factors that may affect the scores of maternal knowledge and concept dimensions. As the age increases, the scores of knowledge and concept dimensions are higher. The average score of pregnant women aged 20 to 24 is 10.06 points. While the average score of pregnant women aged 35 and above was 11.08 points, and the scores of pregnant women of different age groups were statistically different (*PP* < 0.05). Economic income has a significant impact on the scores of the knowledge and ideal dimensions. With the increase of economic income, the scores of pregnant women in this dimension increase (*P* < 0.05). The scores of pregnant women who participated in the maternity school were significantly higher than those who did not participate in the maternity school (*P* < 0.05). There were no statistically significant differences in the scores of maternal knowledge and concepts of different education levels and different pregnancies (*P* > 0.05). The effect of online courses on maternal and child health is shown in Figure 6.

Multivariate linear regression analysis is performed on the factors that may be meaningful (*P* < 0.1) in the single factor analysis. Multicategorical variables enter the regression equation in the form of dummy variables. The results showed that three variables, age, income, and participation in maternity school, entered the regression equation. The scores of pregnant women aged 35 and above were significantly higher than those of 20–24 years old (*P* < 0.05). The scores of pregnant women with economic income between 2000 yuan/month and 4999 yuan/month were significantly higher than those with economic income<2000/month (*P* < 0.05). The scores of pregnant women who did not attend maternity school were significantly lower than those of women who regularly attended maternity school (*P* < 0.05). There was no significant difference between the scores of women who occasionally attended maternity school and those who regularly participated in maternity school (*P* > 0.05). The influence of maternal education on maternal and infant health is shown in Figure 7.

### 5.3. The Mastery of Basic Maternal and Infant Health Skills of Pregnant Women and Analysis of Influencing Factors

A survey on the mastery of the basic skills dimension of maternal and child health of pregnant and lying-in women found that the overall mastery of this dimension is relatively good, and only the mastery rate of “the treatment of abnormal nipples” is below 80%. The highest mastery rate is “breastfeeding skills”, with 457 pregnant women expressing mastery, with a mastery rate of 91.95. The second is “the content and methods of family guardianship”. 427 pregnant women said they had mastered it, and the mastery rate was 85.92%.

A one-way analysis of variance was performed on the factors that may affect the scores of the basic skills of maternal and child health of pregnant and lying-in women. The results showed that there were statistical differences in the scores of pregnant women of different age groups (*P* < 0.05). The women aged ≥35 years old had the highest scores, and those aged 20–24 years old had the lowest scores. The differences in the scores of pregnant women with different economic incomes in this dimension are statistically significant (*P* < 0.05). The women with economic income ≥5000 yuan/month have the highest score, and those with economic income<2000 yuan/month have the lowest score. Participation in the maternity school has an impact on the score of this dimension.  Figure 8 shows the scores of maternal basic skills dimensions.

The factors that may be meaningful (*P* < 0.1) in the univariate analysis were subjected to multiple linear regression analysis. Four variables, age, education level, economic income, and participation in maternity school, were entered into the regression equation. The scores of pregnant women aged 25–29 years in this dimension were significantly lower than those of women aged 20–24 years (*P* < 0.05), and women aged 35 and above scored significantly higher than those aged 20–24 years (*P* < 0.05). The scores of pregnant women with college education and above were significantly higher than those with junior high school education and below (*P* < 0.05). The scores of pregnant women with economic income of 2000–4999 yuan/month (*P* < 0.05) and more than 5000 yuan/month were significantly higher than those with economic income of less than 2000 yuan/month (*P* < 0.05).

## 6. Conclusion

The results of the one-way analysis of variance showed that as the age increased, the scores of the knowledge and concept dimensions were higher. Economic income has a significant impact on the scores of the knowledge and ideal dimensions. With the increase of economic income, the scores of pregnant women in this dimension increase (*P* < 0.05). The scores of pregnant women who participated in the maternity school were significantly higher than those who did not participate in the maternity school (*P* < 0.05). There were no statistically significant differences in the scores of maternal knowledge and concepts of different education levels and different pregnancies (*P* > 0.05). There are statistical differences in the scores of pregnant women of different age groups in this dimension (*P* < 0.05). The women aged ≥35 years old have the highest scores, and those aged 20–24 years old have the lowest scores. The differences in the scores of pregnant women with different economic incomes in this dimension are statistically significant (*P* < 0.05). The women with economic income ≥5000 yuan/month have the highest score, and those with economic income<2000 yuan/month have the lowest score. Participation in the maternity school has an impact on the score of this dimension. The average score of pregnant women who regularly attend the maternity school is 95 points, the average score of pregnant women who occasionally participates in the maternity school is 90 points, and the average score of pregnant women who do not participate in the maternity school is 80 points; the difference is statistically significant. Multiple linear regression analysis found that age, education level, economic income, and participation in maternal school are the influencing factors of maternal basic skills dimension scores.

## Figures and Tables

**Figure 1:** Social support received by users of WeChat parenting group.

**Figure 2:** System overall architecture diagram.

**Figure 3:** Schematic diagram of system front-end functions.

**Figure 4:** Sources of information on pregnant women's health during pregnancy.

**Figure 5:** Awareness of maternal knowledge and concepts.

**Figure 6:** The impact of online courses on maternal and infant health.

**Figure 7:** The impact of maternal education on maternal and infant health.

**Figure 8:** Maternal and child health basic skills scores.

**Table 1:** Participation of pregnant women in school education for pregnant women (*n* = 800).

Attend a maternity school	Number of people	Composition ratio (%)
Participate regularly	100	12.5
Participate occasionally	200	25
Never participated	500	62.5
Total	800	100

## Data Availability

The data used to support the findings of this study are available from the corresponding author upon request.
